The article "Socio-Emotional Wealth, Innovation Environment, and Innovative Investment Path of Family Enterprises: Implications for Environmental Accountability" was published in 2022. Journal: J Environ Public Health.

# Socio-Emotional Wealth, Innovation Environment, and Innovative Investment Path of Family Enterprises: Implications for Environmental Accountability

**DOI:** 10.1155/2022/3759456

**Published:** 2022-07-18

**Authors:** Hui Liu

**Affiliations:** Huzhou Vocational and Technical College, Huzhou 313000, China

## Abstract

Driven by social development, family enterprises continue to grow in terms of scale and number, becoming an important force that promotes China's economic development, and how to achieve the healthy growth of family enterprises has become an inevitable topic. With the increasingly fierce market competition, more and more family businesses have changed from a single market model to cross-industry operation, trying to seek new growth points through industry diversification. Multiculturalism is the product of a particular era, and it is closely related to the great changes in society in a specific era, including new changes in the fields of family, marriage, religion, education, and race relations and even to the international context. Multiculturalism is a theoretical response to these changes and represents the current cultural research tendencies of the international academic community. Socio-emotional wealth and an innovative environment are particularly important for family businesses in a multicultural context. The article first introduces the social emotional wealth and the innovation investment of family enterprises, then focuses on the impact of the innovation environment on the innovation investment of family enterprises, and analyzes the influence mechanism of social emotional wealth and innovation environment on family innovation investment, so as to put forward corresponding countermeasures and suggestions, which also has certain guiding significance for the innovation management and practice of Chinese family enterprises.

## 1. Introduction

In the past, the development of traditional family enterprises only paid attention to the economic development of the enterprise, but ignored the responsibility of family enterprise management to the natural environment. Today's family businesses recognize that economic development is built on environmental sustainability. Therefore, family enterprises now focus on the construction of environmental protection, energy saving, and sustainable development of the enterprise construction. So, this article for environmental responsibility is inspired by the essence of the world.

Multiculturalism refers to the fact that in the case of increasingly complex human society and more developed information circulation, the renewal and transformation of culture are also accelerating, the development of various cultures is facing different opportunities and challenges, and new cultures will emerge in an endless stream. Under the modern complex social structure, we inevitably need a variety of different cultures to serve the development of society, and these cultures serve the development of society, which creates cultural pluralism, that is, multiculturalism in a complex social context.

The article "Socio-Emotional Wealth, Innovation Environment, and Innovative Investment Path of Family Enterprises: Implications for Environmental Accountability" was published in 2022. Journal: J Environ Public Health.

Innovation is an important measure for enterprises to cultivate sustainable competitive advantages, which is of great significance for the sustainable growth and prosperity of enterprises. With the continuous advancement of innovation-driven development strategy and “double creation” strategy, the position of innovation in enterprise development strategy has become increasingly prominent, and the enthusiasm for innovation in the market has reached an unprecedented height. However, family businesses, as an important force in maintaining China's rapid economic growth, generally have the problem of insufficient investment in innovation [1]. Therefore, the exploration of the innovation investment orientation of family enterprises has become a hot topic of academic attention. Drawing on the research of previous scholars and combining it with the content to be studied, this paper defines a family enterprise as follows: (1) the actual controller of the enterprise is a natural person or family; (2) the actual controller directly or indirectly holds the shares of the enterprise and is the largest shareholder of the enterprise.

The existing literature mainly explores the motivation of family enterprise innovation investment from the perspective of resource basis theory, agency theory, and housekeeper theory. However, traditional economic theory is not fully applicable to the study of family business management, and it is easy to contradict theory and practice [2]. In 2007, Frezatti et al. first proposed a theory unique to the field of family business, social emotional wealth [3]. The theory holds that in addition to economic goals, families tend to attach great importance to the protection and development of noneconomic goals such as family control, social relations, and intergenerational inheritance. Since the theory of social emotional wealth was proposed, it has gradually become an important direction to explore the driving force of innovative investment in family enterprises based on this theoretical perspective. The profit and loss of social emotional wealth are an important decision point for family businesses to increase investment in innovation. For example, Radke believe that family businesses will show a tendency to risk aversion in order to protect social emotional wealth, thereby reducing investment in innovation [4]. In addition, Yan Ruosen and Xiao Sha found that family businesses reduce innovation investment in order to maintain close social relations and avoid loss of social and emotional wealth [5]. However, some studies have shown that protecting social emotional wealth does not always reduce the intensity of innovation investment in family businesses. Family businesses will increase their investment in innovation in order to preserve and perpetuate their socio-emotional wealth [6].

The article "Socio-Emotional Wealth, Innovation Environment, and Innovative Investment Path of Family Enterprises: Implications for Environmental Accountability" was published in 2022. Journal: J Environ Public Health.

What is the impact of family protection of social emotional wealth on the innovation investment of family enterprises? Although previous literature has emphasized the importance of family motivation for protecting social emotional wealth in the decision-making of enterprise innovation investment, the influence mechanism of social emotional wealth on the innovation investment of family enterprises has been less deeply revealed and verified. At the same time, social emotional wealth is a multidimensional concept, and most of the existing literature does not subdivide it, thus ignoring the differences in the impact of different dimensions of social emotional wealth on the investment of enterprise innovation. Therefore, this paper will further refine the social emotional wealth and explore the differentiated characteristics and direct effects of its various dimensions on the innovation investment of family enterprises. This research is conducive to further expanding and enriching the research results of family enterprise innovation and also has certain guiding significance for the innovation management and practice of Chinese family enterprises.

## 2. Social Emotional Wealth and Family Business Innovation Investment

### 2.1. Social and Emotional Wealth

#### 2.1.1. The Meaning of Social Emotional Wealth

Social emotional wealth comes from Louis A. Thompson, dean of Arizona State University's Business School. In a 2007 study of the decision-making behavior of more than 1,200 family businesses in Spain, Gomez-Mejia proposed that family businesses have intangible wealth, that is, social emotional wealth (SEW), in addition to economic wealth [7].

As shown in Figure 1, social emotional wealth is the most differentiating factor between family business and other forms of organization. Essential characteristics refer to the noneconomic benefits that families receive from family businesses by virtue of their status as owners, decision makers, and managers. This noneconomic interest covers a wide range of issues, including family control over business, family members' identification with business, close social ties, emotional attachment between family members, and intergenerational family inheritance [8], as seen in Figure 2. When strategic decisions have the potential to threaten a family's existing social emotional wealth, they are motivated by an aversion to the loss of socially affective wealth. Family decision makers will avoid adopting this strategy. Therefore, many scholars have also pointed out that the attitude of family businesses to R&D and innovation activities will be affected by the family's pursuit of social emotional wealth.

The article "Socio-Emotional Wealth, Innovation Environment, and Innovative Investment Path of Family Enterprises: Implications for Environmental Accountability" was published in 2022. Journal: J Environ Public Health.

#### 2.1.2. Social and Emotional Wealth and Innovative Investment in Family Businesses

First, the family's quest for corporate control limits the R&D and innovation activities of the family business. Maintaining family control over the business is often seen as central to the emotional wealth of society. On the one hand, domestic family businesses have long had traditional “home culture” influence, and family control has also received more attention from the family. On the other hand, other dimensions of socio-emotional wealth also need to rely on family control over the business to be realized. For example, leaders who value family obligations often provide family businesses to family members indiscriminately. Family provides employment opportunities through family business resources and provides better working and living conditions for family members. And only by gaining a high degree of control over the enterprise can these benefits be obtained without hindrance. The more a family places control over a business, the more cautious it will be about investing in innovative activities. On the one hand, external funding from innovation and R&D activities can weaken family control over business ownership. R&D activities often require large and ongoing capital investments, and the addition of external investors dilutes the family's control over the business and makes new claims for the strategy, use of funds, and day-to-day management of the business. On the other hand, innovation and R&D activities often require talents with specialized knowledge and advanced skills, and the addition of these talents may also threaten the family's actual management control of the enterprise. Introducing professional talents often increases the organizational structure and management of the authorization requirements, thereby reducing the family's management control over the corresponding R&D departments and technical departments. Therefore, when the family pursues a high degree of control over the enterprise, in order to maintain its ownership and management of the family business, it will avoid risks and try to avoid obtaining external funds or appointing family members as important managers in the long term. These factors also limit the investment of enterprises in innovation and R&D activities.

The article "Socio-Emotional Wealth, Innovation Environment, and Innovative Investment Path of Family Enterprises: Implications for Environmental Accountability" was published in 2022. Journal: J Environ Public Health.

Second, in the process of intergenerational succession, especially in the early stages of the succession process, the willingness of family companies to carry out innovative R&D activities is also weakened. In order for the inheritance to proceed smoothly, it has corporate control and management. The whole family tends to avoid the risks of intergenerational succession. At that time, most of the senior managers in the enterprise are prone to distrust the second-generation successor, making it difficult for the second generation to show its influence on the enterprise [9]. At that time, the second generation tends to pay more attention to the current interests and short-term performance of the enterprise, expecting to make certain achievements and establish their authority in the short term. R&D itself is long-term and highly uncertain, so family businesses try to avoid such uncertainties.

In addition, the pursuit of social ties, especially political relations, by family-owned enterprises can sometimes be a factor in reducing their innovative R&D activities. Because family businesses establish political ties, they are more likely to obtain the protection of local policies, and even if they do not carry out innovative activities, they can maintain a high market share, thereby weakening the stimulating effect of market competition on the innovation of family enterprises. Moreover, when firms reap lucrative returns through political connections, they tend to squeeze investment in other areas, especially in innovation and R&D, and inject resources into maintaining political ties. The research is conducive to further expanding and enriching the research results of family enterprise innovation and also has certain guiding significance for the innovation management and practice of Chinese family enterprises.

### 2.2. Family Businesses

#### 2.2.1. The Meaning, Advantages, and Disadvantages of Family Business

American scholar Gersick has made ownership a watershed between family businesses and nonfamily businesses. Donckels and Frohlich propose that only businesses with more than 60% ownership by family members can be called family businesses. Some scholars believe that family management control is the essence of family business; that is, a family or multiple families with close ties directly or indirectly control the operation of a certain enterprise. Some scholars also consider various aspects of ownership and operational control. For example, the American scholar Chandler defined a family business in his masterpiece “The Visible Hand” in 1987 as follows: the founder and its closest partners (and family members) have always held a majority of the equity, they have strong ties with managers, and they retain management decision-making power. Pan Bisheng regards family ownership as a necessary condition and distinguishes between different stages of development of family businesses by the degree of ownership of management rights. Based on the characteristics of intergenerational inheritance, some scholars believe that “passability” is the key to defining family businesses. When defining what a family business is, Yin Zuoliang and others deliberately emphasize the legal inheritance of corporate ownership, control, and residual claims within the family. A company is a family business when family members own a majority stake, participate in management, form part of a board of directors, and wish to pass the company on to future generations.

The article "Socio-Emotional Wealth, Innovation Environment, and Innovative Investment Path of Family Enterprises: Implications for Environmental Accountability" was published in 2022. Journal: J Environ Public Health.

The private economy of family enterprises is an important part of China's nonpublic economy, and private enterprises provide important support for the rapid development of China's economy [10]. As the owners of family businesses, family members participate in business management. On the one hand, this can reduce the separation of powers and alleviate agency problems. On the other hand, family members will show a tendency to avoid risks when making decisions out of the protection of family wealth and may reject valuable projects when faced with risky or uncertain opportunities. The participation of family members in business management is a “double-edged sword,” which not only can have a positive impact on the family business, but also may lead to the family business becoming self-contained, as seen in Table 1.

A typical feature of a family business is the high level of involvement of family members in the management of the business [11]. As a group closely related to the interests of the enterprise, family members participate in corporate governance to a higher extent. On the one hand, they can reduce the problem of agency in corporate governance, but on the other hand, because family managers are inferior to professional managers in terms of management knowledge and management experience, there are more concerns about the management process, as they may make some conservative decisions that are not conducive to the development of enterprises.

The advantage of family members managing the enterprise is to have a better understanding of the enterprise and to alleviate the agency problems caused by the separation of the two powers of the enterprise, thus promoting the business performance of the enterprise. For small- and medium-sized family enterprises, family management can reduce agency costs and improve execution efficiency, thereby having a positive impact on the value of enterprises. When enterprises are in an industry with fierce competition, family management has a greater positive impact on the value of small- and medium-sized family enterprises.

The article "Socio-Emotional Wealth, Innovation Environment, and Innovative Investment Path of Family Enterprises: Implications for Environmental Accountability" was published in 2022. Journal: J Environ Public Health.

## 3. The Meaning of Family Business Innovation

Innovation is an important driving force for economic growth and social progress, and enterprises occupy a dominant position among the participants in innovation. More and more family businesses have developed and grown, which can inject a steady stream of vitality into China's economic development, provide many high-quality jobs for the society, and have important significance for the development of the country and society [12] After the “innovation-driven development” strategy was proposed in China, China's family enterprises responded to the call of the state, actively carried out enterprise innovation activities, and strived to improve their scientific and technological strength and market competitiveness. The innovative activities of family enterprises can contribute to the high-quality development of China's economy and cultivate more outstanding technologies and talents for practical production and application for the society.  Figure 3 shows that family businesses have some significant management characteristics compared to other types of businesses. For example, the capital of a family business is mainly controlled by a family, the main leadership positions of the family business are held by family members, the management and management rights of family businesses are controlled by family members, and the power and resource allocation of enterprises are guided by blood relations.

Innovation investment shows the willingness and ability of enterprises to innovate and is the manpower invested by enterprises to achieve innovation.

Increasing material and financial resources is the premise of realizing technological innovation and product innovation. Schumpeter pointed out that innovation input is the key for enterprises to obtain competitive advantages, and realizing benefits is enterprise innovation. Schumpeter pointed out that innovation investment is the key for enterprises to gaining competitive advantage, and achieving benefits is enterprise innovation.

The main reason for the investment: from the perspective of investment theory, Zhong Teng proposed that, compared with traditional investment, innovative investment has three characteristics: one is the high sunk cost and adjustment cost, the second is the high risk, and the third is the long cycle. These characteristics make investment in innovation require not only the innovative spirit of managers, but also the company's sufficient funds to support innovative activities. Compared with nonfamily enterprises, the investment in innovation of family enterprises mainly comes from themselves, coupled with the high level of innovation activities, as shown in Figure 4. The characteristics of risk and long cycle make family businesses quite limited in their investment in innovation.

The article "Socio-Emotional Wealth, Innovation Environment, and Innovative Investment Path of Family Enterprises: Implications for Environmental Accountability" was published in 2022. Journal: J Environ Public Health.

Promoting the innovation of domestic enterprises and realizing the transformation of enterprise growth from epitaxial “quantitative” growth to endogenous “qualitative” mode require not only state-owned enterprises to play a “bellwether,” but also a wide range of innovative activities in private enterprises to achieve the healthy and balanced development of social innovation. Family businesses are an indispensable and important part of the private economy. The rapid development of China's real economy is also inseparable from the contribution of family enterprises.

## 4. The Innovation Environment

### 4.1. The Meaning of the Innovation Environment

The concept of Innovation Milieu was first proposed by the Regional Economic Research School represented by the European Innovation Environment Research Group, which emphasizes the synergy between the main and collective efficiency of innovation in the industrial zone and the innovation behavior. The innovation environment should include hardware infrastructure and related soft factors [13], and the innovation environment, as the basic support of the innovation system, plays a very important role in improving the efficiency of innovation. In addition to considering the most basic economic environment, the innovative environmental indicators in the early studies focused on infrastructure factors. Recently, information infrastructure has been increasingly embraced by the scope of the innovation environment [14], and financial development has been included in the innovation environment as shown in Figure 5 [15].

The innovation environment is an external driving force that stimulates the innovation vitality of enterprises and promotes the investment of enterprise innovation. However, in the period of economic transition, due to the different macroeconomic conditions, market demand potential, and institutional and cultural backgrounds of different regions, the innovation environments of various provinces and cities in China are very different.

Cai Xiuling believes that the innovation environment is an institutional factor that provides various opportunities and political guarantees for innovative activities. It is a general term for national policies and regulations, management systems, markets, and services. Foreign scholar Adalot believes that the constituent factors of the innovation environment are the institutions, rules, and practices in the region, which are used to coordinate the inputs and outputs of various innovators in the region. This idea is similar to the idea expressed by Marc Granovet, a sociologist at Stanford University in the United States; that is, economic action is deeply rooted in social action. Both reflections focus on the innovation system rooted in the specific innovation environment. After synthesizing domestic and foreign literature and the research objectives of this article, I believe that the content of the innovation environment should cover factors such as the main body, the management system, the service system, and the cultural atmosphere in which it is located. For these concepts, the universally accepted explanation is the “innovation environment” proposed by Fromhold in 2004. First, the innovation environment is a social contract that encompasses all informals. It is also a network that promotes mutual trust and support and strengthens communication to innovate new products. Second, because it is limited by the spatial distance of the actor, the speed of material circulation is fast and people communicate closely, thus achieving a more efficient rate. Beyond that, the innovation environment is both inside and outside. This overlay will further stimulate consistent behavior between subjects.

The article "Socio-Emotional Wealth, Innovation Environment, and Innovative Investment Path of Family Enterprises: Implications for Environmental Accountability" was published in 2022. Journal: J Environ Public Health.

### 4.2. Identification of the Innovation Environment

According to the European Research Group on the Environment for Innovation (GREMI), companies can be seen as products of the environment and as places where innovative companies are nurtured. The environment is necessary for innovation, and technical know-how, local linkages and local inputs, proximity to the market, and access to high-quality labor in the environment are all factors that determine regional innovation. Together with other enterprises, training centers, technology transfer centers, and local authorities, enterprises should use the resources of the environment to jointly produce new forms of localized production organizations and create an environment conducive to innovation.

GREMI identifies the innovation environment in five ways:

1. The external image of the innovation environment is reflected through the actors, social perceptions, and enterprises and institutions in a certain area.
2. The innovative environment has its internal expressive logic, that is, the self-organization process of human resources. Homeland is structured according to the specialization and functionalization of integration. Micro, meso, and macro levels are coordinated.
3. In the collaborative process of innovation environment, non-economic market areas must be expanded. At the same time, the synergy of the environment is also manifested in the diffusion of innovation.
4. Innovation environment provides an environment for common learning. In the process of common learning, the self-development logic of different innovative operation schemes has been formed.
5. Innovation networks require integrated and flexible specialization. Form a network of strategic alliances and SMEs that are interdependent locally, as well as a network of innovation levels.

The article "Socio-Emotional Wealth, Innovation Environment, and Innovative Investment Path of Family Enterprises: Implications for Environmental Accountability" was published in 2022. Journal: J Environ Public Health.

GREMI expands the environment of innovation from a relatively small community to a region; an environment of innovation is related not only to science and technology themselves, but also to sociocultural ideas. And the exchange of information and knowledge is disseminated not only through material means (communication and computer networks) but also, importantly, through informal and “invisible” chains such as human-to-human contact. The innovation environment is related not only to market space and production space but also to support space. All of this provides new ideas for creating an innovative environment.

### 4.3. Research on the Innovation Environment

For the innovation environment, scholars and experts at home and abroad have done certain research, and the collaborative innovation environment includes a variety of factors that can affect the occurrence of the entire collaborative innovation activity. Current research focuses on how to build an innovation environment and what impact it will have on collaborative innovation.

In terms of the definition of the innovation environment, at present, the academic community has not yet formed a unified definition of the concept of the innovation environment, which was first proposed by GREMI; it is defined as the external environment in which various innovative subjects can cooperate with each other in the complex social relationship of improving the ability of technological innovation [16]. Camagni argues that the innovation environment is one that encompasses local production systems, the various actors involved, and the influence of their industrial cultures, which together interact with markets, cooperation, or networks, resulting in a localized and ever-changing process of learning together [17]. StorDer believes that the innovation environment is a combination of institutions and various rules, and the external environment composed of this combination has a certain role in promoting the mutual cooperation and mutual learning. In China, Jia Yanan defines the innovation environment as an external environment such as material and cultural environment that can support the region's desire to obtain stronger development capabilities, so that all innovative entities can better develop together and form a relatively stable external environment. Huang Qiaoqing believes that the innovation environment is based on the unique current situation in China and that the innovation subject can pass the constraints of the policies, systems, and external environment that can coordinate the common development of various innovative subjects [18]. Cai Xiuling defines the innovation environment as the policy environment including laws and regulations, the current management system, and the economic market and service environment, which can provide rule support and institutional structure support for innovation activities. Through the combining of relevant literature, we can find that the basic agreed definition of the innovation environment and the external environment required by each participant in innovation can effectively play its role and promote the cooperation between the innovative subjects, which can provide important support for the overall collaborative innovation as shown in Figure 6.

The article "Socio-Emotional Wealth, Innovation Environment, and Innovative Investment Path of Family Enterprises: Implications for Environmental Accountability" was published in 2022. Journal: J Environ Public Health.

In terms of the interaction between the innovation environment and the performance of collaborative innovation, different scholars have also adopted different methods and conducted a series of studies based on different levels. For example, Zhao Fumin divided the innovation environment into two types: government-led and market-oriented. After sorting out and normalizing the relevant scientific and technological statistics, the data of the innovation environment and innovation performance were returned to the panel, and a series of evaluations and analyses were carried out on the relationship between the two according to the different situations of the empirical results [19]. Zhang Lijun constructed a regression model after analyzing the innovation environment and the current situation of innovation capabilities and analyzed the impact of the innovation environment on innovation capabilities, indicating that market demand is the factor that can most affect regional innovation capabilities at this stage. Zhou Xuerong measured the innovation efficiency by the Malmquist index method, conducted a regression analysis of the innovation efficiency based on the panel data of the innovation environment for four years, and found that the innovation environment has a great impact on the innovation efficiency of high-tech enterprises. Wang Peng used Moran's I index method to conduct a spatial autocorrelation test on the innovation environment and innovation input, and the results showed that indicators such as loan balances of financial institutions had obvious positive effects on the overall innovation efficiency. Wei Xinxin used interaction term models and panel data to study how the innovation environment plays a role in the performance of high-tech industries.

The article "Socio-Emotional Wealth, Innovation Environment, and Innovative Investment Path of Family Enterprises: Implications for Environmental Accountability" was published in 2022. Journal: J Environ Public Health.

Through the collation of relevant literature, we can see that when studying the current situation of the innovation environment, scholars from different disciplines use different methods to construct relevant index systems according to their actual needs. In the evaluation of collaborative innovation performance in the innovation environment, the most representative source is the “China Regional Innovation Capacity Report,” but the report does not clearly fix the specific indicators at each level of the innovation environment. As is shown in Figure 7, at present, most scholars rely on the content of the report on the construction of the innovation environment, combined with the actual situation, to build their own innovation environment levels and specific indicators at each level. On this basis, the relationship between the two was studied using different evaluation methods. It can be seen that it is necessary to select appropriate indicators and appropriate methods to conduct a series of analyses of the impact of the innovation environment on the performance of collaborative innovation.

### 4.4. Innovation Environment and Innovation Input of Family Enterprises

Research shows that when the survival and development of family enterprises are threatened, they will improve their risk tolerance and increase investment in enterprise innovation, so as to establish competitive advantages through innovation and realize long-term survival of enterprises, so as to protect the economic and emotional wealth of the family [20].

Based on the analysis of the previous article, the profit and loss of social emotional wealth is an important decision point for family enterprises to increase innovation investment. However, the strategic decisions of enterprises are the result of a combination of internal and external environments, and differences in external environments can lead to differences in the social emotional wealth [21], which in turn makes the level of innovation investment of family enterprises different. In areas with a poor innovation environment, family businesses often face problems such as insufficient innovative talents, single financing channels, and imperfect legal environment, which will increase the risk of enterprise innovation activities. In this case, in order to avoid the loss of social emotional wealth, the family business will reduce the investment in innovation. On the contrary, in a good innovation environment, the market generally has a sound legal environment and a sound financial and taxation system and gathers a large number of outstanding talents. At the same time, enterprises have more independent choices and can choose their preferred projects according to market demand for innovative investment. In this scenario, the risk of loss of social emotional wealth caused by the company's innovation will be greatly reduced, which will help promote the family business to increase innovation investment. In addition, studies have shown that when the survival and development of the enterprise are threatened, the family business will increase the risk tolerance and increase the level of investment in corporate innovation [22], in order to establish a competitive advantage through innovation, achieve long-term survival of the enterprise, and thus protect the family's economic and emotional wealth.

The article "Socio-Emotional Wealth, Innovation Environment, and Innovative Investment Path of Family Enterprises: Implications for Environmental Accountability" was published in 2022. Journal: J Environ Public Health.

## 5. Conclusions and Policy Recommendations

Family businesses are a complex of interactions and connections between families and businesses, and their innovation inputs weigh not only economic, but also noneconomic goals. This paper examines the impact of social emotional wealth and innovation environment on the innovation investment of family businesses in a pluralistic context. The results show the following: (1) the impact of different dimensions of social emotional wealth on the innovation investment of family enterprises is different; (2) the innovation environment of the region where the family enterprise is located will also have an impact on the innovation investment of family enterprises.

Based on the research conclusions, this paper puts forward the following policy recommendations: (1) China's family enterprises should be aware of the dual impact of social emotional wealth on the innovation investment of family enterprises, in order to minimize the negative effect of social emotional wealth, and cannot blindly reduce the intensity of innovation investment in order to maintain family control and family identity, which will directly affect the transformation and upgrading of family enterprises and long-term development. (2) In the special period of transformation, family enterprises should establish good ties with the government, which helps enterprises to grasp the market trend in a timely manner and obtain certain indispensable key information and resources, thereby reducing the risk of family enterprise innovation activities and promoting enterprises to improve the level of innovation investment. (3) Family enterprises should strengthen the cultivation of second-generation capabilities and qualities and, at the same time, appropriately allow second generation to enter the enterprise as soon as possible, giving them sufficient time to contact corporate governance and accumulate management experience, so as to give full play to the positive role of intergenerational inheritance in enterprise innovation investment. (4) The innovation environment is an external driving force that enterprises cannot ignore to carry out innovation activities. The government should establish a market environment of fair competition and sound laws and regulations and give full play to the role of market mechanisms in allocating innovative elements. At the same time, it should strengthen the effectiveness and transparency of policies, standardize the incentive mechanism for innovation, and improve the innovation network system, so as to create a market environment conducive to the innovation of family enterprises, remove obstacles to the external development of family enterprises, and enhance the innovation power of family enterprises.

The article "Socio-Emotional Wealth, Innovation Environment, and Innovative Investment Path of Family Enterprises: Implications for Environmental Accountability" was published in 2022. Journal: J Environ Public Health.

## Figures and Tables

**Figure 1:** Distribution of the world's top 100 oldest family businesses.

**Figure 2:** Age distribution of family business leaders.

**Figure 3:** Family businesses.

**Figure 4:** Example of family business investment.

**Figure 5:** Family business industry distribution.

**Figure 6:** The family business inheritance plan.

**Figure 7:** Business incubators.

**Table 1:** Financial and nonfinancial objectives of family businesses.

Financial and nonfinancial objectives of family businesses	
Financial objectives (economic efficiency)	Nonfinancial goals (socio-emotional gains)
Maximizing profits (shareholder returns)	Creating and protecting the family's spiritual wealth
Sales revenue	Showing family prestige
Profits	Continuing family values
Market share	Continuing the influence of family social status
Rapid growth and scale expansion	Meeting the family's emotional homecoming needs
Getting bigger and stronger fast	Planting deeper, living longer

## Data Availability

The labeled data set used to support the findings of this study is available from the author upon request.
